# Awareness of Prostate Cancer among the Sportsmen in the Republic of Serbia

**DOI:** 10.1155/2022/8400768

**Published:** 2022-11-16

**Authors:** Tamara Panajotović, Nikola Panajotović, Milos Vukcević, Aleksandra Dragicevic, Iva Vojinović, Sladjana Kovacević, Mina Dimitrijević

**Affiliations:** ^1^University of Belgrade, Faculty of Organizational Sciences, Belgrade, Serbia; ^2^General Hospital Pančevo, Pančevo, Serbia; ^3^University of Mediterranean in Podgorica, Faculty of Law, Podgorica, Montenegro; ^4^University of Belgrade, Faculty of Mechanical Engineering, Department for Biomedical Engineering, Belgrade, Serbia; ^5^University of Belgrade, Faculty of Medicine, Belgrade, Serbia; ^6^University of Belgrade, Faculty of Special Education and Rehabilitation, Belgrade, Serbia

## Abstract

Prostate cancer is the second most commonly occurring cancer in men. Regardless of statistics, screening for prostate cancer is an individual decision and most male patients come for their first examination with an already developed disease, as they are not adequately informed. The study aimed to emphasize the importance of preventive tests for urological diseases in the Republic of Serbia, raise awareness about urinary problems, and present social marketing strategies for prevention. The results confirm the generally lower awareness of respondents under the age of 30, followed by those who finished university, go to the doctor two or three times a year, and receive information other than by watching TV. Implemented research indicates the influence of the marketing principles and social marketing strategies on possible target groups of the male population over 50, which is aimed at raising awareness of the importance of prevention of urological diseases and the expected changes in the health behavior of the target population.

## 1. Introduction

According to a major global study on the causes of death and disease, published in the medical journal The Lancet − The Global Burden of Disease, an important barrier to increase life expectancy in every country in the world is cancer. It is the second leading cause of death, with nearly 10 million deaths in 2020 [1]. As a global disease, cancer spreads rapidly, with a prediction estimate of 30.2 million new cases and 16.3 million deaths by 2040 [2, 3].

On the other hand, cancer results in an economic burden on countries, healthcare systems, patients, and their families. This burden refers to healthcare spending and productivity losses from morbidity and premature mortality. Data on the amount of expenditures caused by cancer are unknown; however, some countries have economic analyses that indicate resource allocation decisions and investments in cancer control programs. Mentioned programs include the raising of awareness, prevention, early detection, treatment, survivorship, and end-of-life care. The amount spent on cancer in 2017, in the US, was 1.8% of gross domestic product (GDP), detailed US$161.2 billion; US$30.3 billion, and US$150.7 billion (healthcare, loss in productivity from morbidity, and premature mortality, respectively). Data for the European Union in 2018 show a total burden of €141.8 billion or 1.07% of GDP. The explanation for the mentioned burden lies in healthcare spending of €57.3 billion, productivity losses due to morbidity and premature death, €10.6 billion and €47.9 billion, respectively, and informal care costs of €26.1 billion. In summary, it means that the economic burden of lost productivity due to morbidity and premature death from cancer is nearly 60% of the total economic burden associated with cancer in the European Union countries [4–6]. Intending to tackle this issue, worldwide healthcare systems are facing stiff challenges.

According to existing data, by applying existing evidence-based prevention strategies and avoiding risk factors, between 30 and 50% of cancers can currently be prevented. Screening, early detection of cancer, and appropriate treatment and care of patients can also contribute to reduce the cancer burden since many cancers have a high chance of being cured if they are diagnosed early and treated appropriately [2]. A delay in seeking help for cancer symptoms is the main factor and reason consistently shown to be associated with late diagnosis and treatment [7]. As poor awareness may lead to poor uptake of screening modalities and delay in diagnosis, cancer awareness is the key to early detection and better health-seeking behavior [7].

The emphasis in this paper is on prostate cancer, as the fourth leading cause of death among men, with an estimated almost 1.4 million new cases and 375,000 deaths worldwide in 2020 (Figure 1).

Prostate cancer has been diagnosed in over one-half of the countries of the world (112 of 185) with an incidence rate 3-fold higher in transitioned than in transition countries. The highest rates are found in Northern and Western Europe, the Caribbean, Australia/New Zealand, Northern America, and Southern Africa (around 83.4 per 100,000 men). The new observatory and prediction rate until 2040, based on GLOBOCAN (Figure 2), is 2,29 million new cases with a small variation in mortality rate (an increase of 1.05%) [8–11].

In cancer deaths, the Republic of Serbia is an inglorious leader in Europe. In 2020, out of the population of 8.74 million, 49,043 new cases and 28,107 deaths have been recorded. During 2020, Serbia's prostate cancer mortality rate is ranked third and its incidence rate is ranked fourth, according to the Global Cancer Observatory. It is a malignant disease that affects the male population, and if not detected and treated in time, certainly leads to death. Statistics show that only 40% of patients are detected in the curable phase of the disease. What distinguishes prostate cancer from other malignancies is its slow progression, and medical research indicates that the disease can appear as early as the age of 30 but rarely shows the first signs before the age of 50 (in less than 1%). Most patients develop a clinically detectable form of the disease after the age of 55, and the largest number of patients is in their 60s. It is not known when the disease begins to progress in a person with a clinically nonmanifest (latent) form. The revolution in prostate cancer discovery and treatment began in the late 1980s and 1990s with the discovery of PSA (prostate-specific antigen), whose elevated values in the blood most likely indicate the existence and progression of the disease (levels rise with increasing cancer mass) [12–20].

Usually, patients are unaware that prostate cancer does not cause any complaints until it reaches the preterminal phase and they are not informed that tumor markers (PSA) can help in the early detection of the disease. Descendants of a person who has prostate cancer are at great risk of getting prostate cancer, but in much earlier years, which is another fact unknown to the male population. [15, 17] There is no direct evidence that any form of behavior or adequate nutrition can prevent cancer, which is not a popular belief.

Modern health care policies use social marketing strategies to influence the target group's behavior and promote social welfare activities [21] and in that way, prevent and decrease malignant diseases. As a modern and universal communication tool for influence on urologic diseases, social media is used [22]. Adequate social marketing implementation can increase patients' awareness and the number of preventive examinations that will result in early detection and treatment of prostate cancer and reduce the overall prostate cancer mortality rate [23]. Adequately provided information from the chosen physician can also lead to a greater number of early-detected prostate cancers [24].

Central issues of health policy are related to the development of healthy lifestyles and strengthening the individual responsibility for behavior and attitudes toward health. Healthy, responsible behavior promotion, along with all measures for the healthcare system's development, contributes to eliminating the consequences of risky behavior and reducing population mortality [25].

Adequate social marketing aims to inform the population about preventive examinations that can detect malignant diseases in the early (curable) phase, as well as inform about the symptoms and signs of the disease that should make the patient visit the doctor. Also, adequate social marketing strategies can indicate healthy habits and patterns of behavior, all with the aim of preventing diseases that are the leading causes of illness and death [26–30].

The idea for the research came from the fact that the number of prostate cancer patients in Serbia is increasing, the nonexistent screening program, the sporadic publication of newspaper articles in terms of warning and awareness among the male population, and the overall poor informational status of the population. Another reason for the aforementioned research is the presence of other cancers, with the highest mortality rate, and their visibility at a significantly higher level, both through screening programs conducted by the Institute for Public Health of Serbia “Dr. Milan Jovanovic Batut,” media publication and appearance of the experts in the field.

The main goal of the work was to examine the awareness of adult sportsmen from urban areas in the Republic of Serbia about risk factors, diagnosis, and treatment of prostate cancer and further, based on the results, to indicate possible ways to improve this information. In order to obtain this information, two tests for data analysis were applied in the paper:- *T*-test and ANOVA, all with the aim of checking the set hypotheses. The aim of the present paper is to raise awareness of prostate cancer risks and symptoms and to explain the importance of sportsmen's involvement in informing the population and their call for testing.

## 2. Materials and Methods

The sample involved 98 respondents, sportsmen from urban regions of Serbia for the period July– September 2019: Novi Sad, Belgrade, and Pančevo, using the data collection method PAPI (Paper and Pencil Interviewing)–face-to-face field research in the participants' homes. Of the 15 questions, 8 considered sociodemography and their general attitudes and habits regarding health and 7 were for specific medical conditions. It was created by the authors in collaboration with specialists and experts in the field of urogenital medicine. With the aim of understanding the details of the prevention of urologic diseases and how well patients are informed and instructed after a urological disease is diagnosed, six urologists from the General Hospital of Pančevo were involved.

In order to get one index of awareness about urologic diseases, a couple of steps were performed.

1. Each question from the set regarding specific urologic diseases was recorded depending on what the most accurate answer was (according to urologists). 1 represents that the person is informed, and 0 represents that the person is not informed. Six questions were used in the creation of the awareness index.
2. The sum score was transformed on a scale of 0 to 1, and the new variable representing the awareness index was obtained.

The awareness index is used as a dependent variable, while sociodemographic variables and general variables (Table 1) related to healthcare habits are used as independent variables.

Data were processed in accordance with high standards in order to provide relevant information. The software used for data analysis was IBM SPSS (Version 26.0, Chicago, IL, USA).

Data analysis was done in two phases, which are as follows:

- Descriptive statistics and simple percentage distribution of relevant questions
- *T*-test and ANOVA analyses for comparing awareness about urological diseases among different groups

## 3. Results

In accordance with the obtained study, type of representative, and disease, the obtained results are separated into three tables. The first following, Table 2 shows the frequencies of respondents to each question related to general health care habits. The majority of respondents visit a doctor once a year, mostly for follow-up. The top three resources when finding information about diseases, diagnosis, treatment, and prevention are chosen doctors, doctor specialists, and the Internet. More than 60% of respondents assess their health as good or great, and the largest number of respondents (53.1%) believe that they are superficially informed about urologic diseases.

Table 3 shows the distributions of respondents related to sportsmen included in the awareness index. Two-thirds of the respondents believe prostate cancer occurs frequently or moderately in men. The majority of respondents believe prostate cancer occurs among people older than 50 years. The respondents have divided opinions when it comes to whether prostate cancer has clear symptoms or not. Most of them believe that prostate cancer could be diagnosed and treated and that they themselves should visit doctors preventatively regarding the prostate. People have divided opinions on whether taking supplements for the prostate on time can prevent prostate diseases.

Question 7 from Table 3 shows the distribution of the questions but was not included in the awareness index. A bit more than half of the respondents know what a PSA marker is.

For the sake of better categorization of respondents, we have made a permanent criteria regarding the awareness index score. We have categorized respondents into four groups regarding their awareness index score. Every respondent with a score below 0.4 was defined as “poor awareness,” if a score is in the range of 0.41 to 0.60 was defined as “medium awareness,” if it is in the range of 0.61 to 0.8, it was defined as “good awareness,” and if a score is higher than 0.80, it was defined as “great awareness”.

Table 4 contains descriptive statistics for every independent variable used in research. Regarding age, the highest score we notice in this group is 51 to 60 years old and the lowest with the youngest (20 to 30 years old). If we compare the average scores of the awareness index regarding the education level of respondents, the highest score is noticed with those who finished primary school, those who do not visit the doctor, and those who were informed about the disease through TV.

## 4. Discussion

Modern health care policies use social marketing strategies to influence the target group's behavior and promote social welfare activities [27], and in that way, prevent and decrease malignant diseases. As a modern and universal communication tool for influence on urologic diseases, social media is used [28]. Adequate social marketing implementation can increase patients' awareness and the number of preventive examinations. The main result will be in early detection and treatment, with a reduced overall prostate cancer mortality rate [29]. Adequately provided information from the chosen physician can also lead to a greater number of early detected prostate cancers [30].

Early diagnosis of prostate cancer and every other type of cancer is reflected through a high awareness of cancer. It is strongly emphasized and indicates a certain socially acceptable behavior that supports it. On the other hand, the absence of these patterns and the delay in seeking help are attributed to limiting factors, which include illiteracy, financial limitations, superstition, etc. [7].

An effective prostate cancer prevention strategy would provide many benefits to men with a significant positive impact on public health. The mentioned strategy would have great potential to reduce the high risk of developing prostate cancer and the morbidity associated with cancer treatment. It would be particularly effective in newly diagnosed patients with biologically indolent prostate cancer who are still undergoing therapy with curative intent instead of active surveillance and ultimately, the inability to eradicate life-threatening metastatic prostate cancer. The currently available epidemiological data show that lifestyle has a high role in the factors for the occurrence of cancer, especially if it is considered that prostate carcinogenesis lasts for many decades. In that case, lifestyle modification can be a very good and highly cost-effective way to slow down the development of the disease [14].

The high global incidence of prostate cancer indicates the necessity of strengthening existing tools for the identification of prostate cancer and the introduction of new prevention strategies to reduce the impact of this disease on public health in the future. A positive trend that played a revolutionary role in the diagnosis of prostate cancer is the identification of the PSA biomarker. Since 1980, a double incidence of prostate cancer has been noted in the USA and other countries, especially in the West [14, 31, 32]. However, PSA was not recommended for the screening program due to the relevant overdiagnosis and the severe side effects of treatments.

According to the study obtained by Mohammed Al-Azri et al. [33], similar results were found compared to the presented work. The main reasons for the delay in early diagnosis, as well as poor results, are poor awareness of cancer symptoms and misinterpretation of these symptoms. Studies conducted in Oman have shown a low awareness of carcinoma in general, especially of the symptoms of prostate cancer. The same or very similar findings were reported in other Arab countries (Saudi Arabia, Egypt, and Jordan). In the main conclusion, it could be seen that in addition to their poor knowledge, the fair attitude of the participants toward prostate cancer examination and screening practices was also demonstrated. The study also showed that younger participants had more knowledge about prostate cancer. Based on the conducted research, it was seen that the largest amount of knowledge of the participants are based on the knowledge obtained through social media, which is proof that social media is a part of a new trend in public health education. Also, individuals with a higher level of education and income showed greater awareness of PSA testing and reported attending routine annual examinations [34, 35].

In addition to the abovementioned observations, the results of a large independent survey conducted in six European countries (France, Germany, Italy, Spain, Sweden, and the UK) and the USA clearly show a lack of awareness about prostate cancer, the PSA test, and early treatment among the general population. Out of the total number of people tested, 39% of men and 28% of women had general awareness of prostate cancer, while 97% of respondents said they had heard of the disease when asked directly. What also turned out to be interesting is that men mentioned breast cancer more often than prostate cancer (46% vs. 39%, respectively). Regarding urinary problems, they recognized them as possible symptoms, but very few understood that the disease can be asymptomatic. Also, respondents who stated that they had prostate cancer or that someone from their close or distant environment had a problem had very low knowledge about the PSA test. Regarding the difference in levels of prostate cancer awareness between the countries in the survey, almost twice the difference in the level of spontaneous awareness was observed between men living in Germany and those living in France (54% vs. 29%, respectively). In Great Britain, men and women were equally informed, while in other countries, men were more informed than women. In the end, it can be concluded that the awareness of prostate cancer and the PSA test was almost 3 times higher between the USA and Germany (48% vs. 17%, respectively), as well as between the USA and all six mentioned European countries [36].

The theme of this paper is about awareness and symptoms of prostate cancer among sportsmen, and supporting the data, there is scientific evidence that confirms the claim that women are more concerned about family health. The conducted study indicated faster and better reactions in women in the following aspects of cancer, recognition of early manifestations of various cancers, timely detection of obstacles to seeking help, and timely reporting of perceived obstacles. Women with a higher level of education were ready to face breast and cervical cancer and thus take control of their health. Also, women showed a deep interest in the health of their partners and noticed changes that men themselves did not see in themselves. They have also been proven to play a key role in making decisions in the treatment of their spouse or partner diagnosed with prostate cancer, as well as in screening. However, few studies have been conducted on women's knowledge of prostate cancer, and it is necessary to map the evidence to establish their knowledge as a public health tool to reduce the disease [37–42].

One of the most recent reports about the involvement of sportsmen in prostate cancer awareness [43] was from the UK charity, Prostate Cancer UK, which provides different types of supports for example, for men, funds research, and lobbies for drug availability, as well as many other things. The charity has done great work by implementing public figures to talk openly about their health problems from the beginning of prostate cancer detection throughout the whole healthcare journey. Many of them publicized their diagnosis and persuaded other men to get themselves tested by telling their personal stories. Their involvement and talk had an extremely high impact on public awareness and its raising [43].

Common to all these studies is the need to see the level of information about prostate cancer in terms of its frequency, symptoms, prevention, treatment, and PCA test. A study conducted on 98 athletes confirmed the basic knowledge of the term and indicated that the majority of respondents believe that prostate cancer occurs in people over 50 years old (69.4%). What is worrying is that only a third of respondents are aware that prostate cancer does not always give clear symptoms (33.7%) and that almost half of respondents have never heard of the PCA test (46.9%).

On the other hand, the vast majority are aware that prostate cancer can be diagnosed and treated (86.7%), as well as the positive effect of preventive visits to the doctor (87.8%).

In our study, the majority of men had adequate knowledge about prostate cancer in terms of whether prostate cancer be diagnosed and treated with 86.7% and have the similar value compared with other studies of 82.1% and 64%, respectively [44, 45]. A similar finding has also been observed in another study conducted in Jamaica, with 96% of men correctly responding to questions about prostate cancer [46]. By contrast, in comparison with other studies from different countries, this rate was better than that which has been reported in South Africa (45.7%) among men attending a urologic outpatient clinic [47] and in Uganda (54.1%) [48]. Regarding knowledge of the PSA test, we found that 53.1% had heard of it before, compared to 72.7% and 41.8% [44, 45]. This value is a little bit higher than a survey conducted in Uganda in 2013 reported 52.1% [48]. Amongst the risk factors for developing prostate cancer are being over the age of 50. 69.4% compared to 65.9% [44] of the respondents correctly identified age >50 years.

The major sources of information about the urinary diseases were physicians, the Internet and television, compared to reference [44]. where the major sources of information about the PSA test were physicians, television/newspapers, and family. Men who had received information from a physician were more likely to know about and take up a PSA test [44]. For example, Carrasco-Garrido et al. [49] found that men who had received information from healthcare workers had a higher probability to know about and to receive a PSA test. Also, in another study conducted in the United States of America, the most frequent sources of information were physicians (86%) and mass media (62%). By contrast, in reference [48], only 12.3% of respondents reported that physicians informed them about screening for prostate cancer.

If we look at the descriptive statistics in relation to information about school education and the way from where they got some information, we can see the highest score is noticed with those who finished primary school, those who do not visit doctors, and those who get information about disease on TV. The conducted study based on specially prepared questionnaires indicates that there is no excessive difference in the awareness of sportsmen in the Republic of Serbia in relation to the population in the world.

Also, a shortcoming was seen in terms of the lack of studies that examined the awareness of athletes about prostate cancer. As shown, the athletes were mentioned only through the media, in the form of various newspaper articles and in associations in the framework of the fight against prostate cancer, as well as in personal stories.

With regard to this research and its findings, as well as other mentioned studies, which were done with the aim of discovering the level of awareness, a campaign to promote urological diseases in the Republic of Serbia is suggested. The aim of the campaign would be to raise awareness of urological diseases and to improve the general health of the target population in the Republic of Serbia by using eHealth services, e.g. mobile and web apps. The campaign goal is to decrease the number of urological diseases in the country, and its impact is reflected in the greater understanding of the importance of urological diseases and prostate cancer prevention. It is of paramount importance to state that the campaign should be at the national level. As a result, the campaign would get full media coverage and would become one of the most important strategies. In Serbia, there are the Nation Youth Strategy, the National Cervical Cancer Prevention Program, the National Breast Cancer Early Detection Program, as well as the recently adopted National Program for Safeguarding and Improving Sexual and Reproductive Health. Starting a campaign might contribute to people's being better and more efficiently informed about urinary diseases.

More specifically, by reviewing the literature and talking to athletes, it was seen that athletes and their popularity among the public could be of crucial importance for raising awareness about urogenital diseases, especially with an emphasis on prostate cancer. As we have already mentioned, sportsmen in the Republic of Serbia have not shown an enviable level of information and awareness about prostate cancer. Therefore, we propose the following steps to improve the current situation:

1. Post hashtags on social media (as they are one of the best ways to draw attention to important issues: Facebook, Twitter, Instagram, Snapchat, YouTube, TikTok, etc.)
2. Spread awareness in the workplace (print and distribute guides throughout the place of work to provide colleagues with information on prostate cancer)
3. Attend events (many events are going virtual; a man may also be able to find one that he can join online from the comfort of his own home)
4. Sportsmen can wear shirts with messages that mention prostate cancer
5. Get a prostate cancer screening (one of the best ways men can show support in September-and beyond. It is a great way to take care of your own health while also inspiring other people with prostate problems to do the same.)
6. The takeaway (Raising awareness for prostate cancer is one of the best ways to help people learn about signs, symptoms, and preventive screening. It also helps build communities and foster connections.).

Also, the month of September is the month of fighting and raising awareness about prostate cancer. The very importance of timely prevention and the problem it creates (number of new cases, mortality, reduced awareness) can be concluded by looking at the announcement of the White House on August 31, 2022, “A Proclamation on National Prostate Cancer Awareness Month, 2022”.

The limitations of the study, in this case, are the relatively small number of respondents, which is further reduced when the number is divided within that division into age subgroups and subgroups with regard to educational status. The results obtained in this way represent the beginning of future studies and open the door to research, and on the other hand, the results indicate a lack of knowledge and awareness about prostate cancer. Certainly, in this particular case, they cannot be generalized to the entire adult, urban population since they do not include the other regions of adult population (all big cities, villages, and other country regions); so, a large national study should be done. Also, one of the limitations of the study is the absence of some other factors that could affect the level of information about the considered diseases, e.g., property status, the presence of these diseases in the respondents themselves or their relatives, etc.

## 5. Conclusion

Despite advances in care and the main health priority of stopping cancer, prostate cancer is the most commonly diagnosed cancer in over 50% of countries (112/185), with more than 1.4 million new cases and 375,000 deaths in 2020 alone. The study conducted, as well as public material available through scientific publications, indicates that there is a clear need to improve the basic concepts and general knowledge of both athletes and the general public about the practice of prostate cancer screening. The prostate cancer screening program in the Republic of Serbia does not exist and therefore does not represent an obligation; patients voluntarily go for examinations, which, with this level of general information and awareness, turned out to be very bad. Also, an acceptable level of recognition of risk factors for prostate cancer was indicated, but their recognition of symptoms was below the acceptable limit. The study showed that increasing the awareness of the population, athletes in our case and men globally, is crucial and in this case, is connected with a higher level of education. In accordance with the abovementioned statements, the key next steps in the continuation of surveillance would imply the necessity for doctors to engage more and talk more with their patients in order to provide them with as detailed and accurate information as possible and then refer them to specific examinations and problem-solving. Considering the shortcoming of the study in the number of respondents, in order to confirm the above data, it is necessary to conduct a larger study at the national level. It can also be concluded that the participants used social media the most as a source of information about prostate cancer, and the evidence showed that social media is a powerful tool for increasing community awareness about cancer prevention, screening, and treatment in real life and time. As a unified result of the study, it can be said that it is necessary to conduct more campaigns to raise awareness in the community by including public figures with an apostrophe to professional athletes, role models of the nation, but also famous doctors (urologists), who will indicate problems, symptoms, and methods of diagnosis and treatment. This connection should be established through guest appearances on television shows, followed by the distribution of information leaflets aimed at men and women in certain settings, such as waiting rooms in health centers and urology clinics in hospitals.

## Figures and Tables

**Figure 1:** Schematic presentation–Estimated number of new cases in 2020 in males, worldwide, all ages (source data: https://www.uicc.org/news/globocan-2020-new-global-cancer-data).

**Figure 2:** Estimated number of new cases from 2020 to 2040. Both sexes, age (0–85+) (source data: https://www.uicc.org/news/globocan-2020-new-global-cancer-data).

**Table 1:** Sociodemographic variables–frequencies.

		Frequency in %	Number of cases (n)
*Males (n* *=* *98)*	*Age*		
	20–30	19.4	19
	31–40	22.4	22
	41–50	18.4	18
	51–60	19.4	19
	61–70	12.2	12
	71 and above	8.2	8
	*Education*		
	Elementary school	6.1	6
	High school	52.0	51
	University	41.8	41

**Table 2:** The frequencies of respondents related to general health care habits.

Answers to questions	Respondents (%)
*1. How often do you visit a doctor?*	
Once a year	30.6
2 to 3 times a year	21.4
3 to 5 times a year	11.2
More than 5 times a year	16.3
Do not visit	20.4
*2. I Visit a doctor for*	
Advice	12.2
Follow up	66.3
Yearly check-up	21.4
*3.* I received information about the disease through	
TV	3.1
Internet	16.3
Chosen doctor	49.0
Doctor specialist	26.5
Pharmacist	1.0
Friend	4.1
*4. I Would say that my health is*	
Great	24.5
Good	38.8
Satisfied	30.6
Poor	6.1
*5.*I am informed about urological diseases, treatment, and prevention	
Aware	27.6
Superficially	53.1
Not informed	19.4

**Table 3:** Frequencies of respondents related to prostate cancer.

Answers to questions (correct answer is marked with ^*∗*^)	Respondents (%)
*1. Do you know how often prostate cancer occurs?*	
No	4.1
Rare	13.3
Extremely rare	14.3
Moderate	33.7
Often^*∗*^	34.7
*2. Do you know which age group is the most vulnerable when it comes to prostate cancer?*	
Do not know	29.6
Younger people	1.0
People older than 50 years^*∗*^	69.4
*3. Does prostate cancer have clear symptoms that indicate that the doctor's help is needed?*	
Yes	34.7
No, they are mild so can be overlooked	31.6
No clear symptoms^*∗*^	33.7
*4. Can prostate cancer be diagnosed and treated?*	
Yes^*∗*^	86.7
No	13.3
*5. Do you think it is necessary to visit a doctor preventatively*about the prostate cancer*?*	
Yes^*∗*^	87.8
No	12.2
*6. If I start to take supplements for the prostate on time, can I prevent prostate diseases?*	
Yes	50.0
No^*∗*^	50.0
*7. Have you heard about PSA markers?*	
Yes	53.1
No	46.9

**Table 4:** Descriptive statistics—awareness index by sociodemography and habits and attitudes towards health.

	Mean	Standard deviation
*Age*		
20–30 years old	0.41	0.14
31–40 years old	0.48	0.15
41–50 years old	0.49	0.15
51–60 years old	0.53	0.13
61–70 years old	0.49	0.15
71 and older	0.48	0.17
*Education level*		
Primary school	0.53	0.13
Secondary school	0.50	0.15
University	0.44	0.13
*Frequency of visits to doctor*		
Once a year	0.49	0.14
2 to 3 times a year	0.40	0.12
3 to 5 times a year	0.48	0.14
More than 5 times a year	0.49	0.15
Do not visit	0.53	0.15
*Reason of visits to doctor*		
Advice	0.49	0.13
Follow up	0.48	0.15
Yearly checkup	0.47	0.12
*Source of information about disease*		
TV	0.61	0.25
Internet	0.44	0.17
Chosen doctor	0.48	0.13
Doctor specialist	0.49	0.14
Pharmacist	0.50	
Friend	0.50	0.19
*Perception of personal health*		
Great	0.47	0.12
Good	0.46	0.16
Satisfied	0.50	0.14
Poor	0.50	0.18

Furthermore, the results indicate that respondents are aware of prostate cancer at a medium level, regardless of their characteristics. The general mean score of the awareness index is 0.48.

## Data Availability

The data used to support the findings of this study are included within the article.
